RETRACTED

# Clustering digital learning pathway preferences from the perspectives of epistemic justification on self-regulated learning, social presence, and resources

**DOI:** 10.1016/j.heliyon.2023.e20038

**Published:** 2023-09-11

**Authors:** Min Lan, Qian Huang

**Affiliations:** a Key Laboratory of Intelligent Education Technology and Application of Zhejiang Province, Zhejiang Normal University, Jinhua Zhejiang 321004, China; b Research fellow, Lee Kuan Yew Centre for Innovative Cities, Singapore University of Technology and Design, 8 Somapah Road Building 3 Level 2, Singapore 487372, Singapore

**Keywords:** Digital learning, Learning preference, Epistemic justification, Self-regulated learning, Social presence

## Abstract

The beliefs about knowledge and knowing have a decisive effect on students' digital learning. Merely using self-reported questionnaire to investigate people's epistemic justifications about digital learning is incomprehension and has its methodological limitations. Therefore, this study used an explanatory sequential design, i.e., clustering followed by content analysis and affective comparisons, to explore people's preference, epistemic justifications, and affective perceptions on digital learning pathways. First, a latent class analysis was conducted to categorise 201 survey participants based on their preferences towards seven types of digital learning pathways. Four clusters were identified. Second, we conducted thematic analysis, relational content analysis and affective analysis on sixteen participants' digital learning experiences. Based on the framework of Internet-based epistemic belief, self-regulated learning, and community of inquiry, three dimensions of digital learning justification were identified, which mutually impact on one another. Furthermore, interviewees' affective perceptions in different clusters were compared, showing different patterns regarding the three dimensions above. These differences informed digital learning designers on instructional designs, teachers' selection of digital learning tools, and policy makers on promoting professional development for digital literacy improving.

## 1 Introduction

Using digital pathways for learning is becoming an indispensable demand for people in the technology-enabled era. Digital learning pathways (DLPs) are self-paced, affordable online learning resources that empower people to learn, such as mobile learning (e.g., using educational apps for learning), MOOCs (e.g., learning systematic knowledge on Coursera), social media (e.g., self-initiated group learning through WhatsApp), and e-Book (e.g., reading a book on Kindle). Compared to traditional face-to-face classroom learning, these DLPs are normally positioned as services for informal learning or non-formal learning, i.e., outside of the traditional learning classroom setting in school.

RETRACTED

However, impacted by the traditional formal learning settings, people may prefer some DLPs to be authoritative resources for systematic learning (e.g., learning on MOOC), while for some other DLPs, people may consider them as tools for leisure-oriented informal learning experiences (e.g., learning something for fun on mobile apps). In this digital era, people have more chances to select the DLPs to satisfy their learning needs. People with more DLPs selecting and using experiences could form their own beliefs towards the values, efficacy, and impacts of digital learning (DL) [1,2]. In turn, the gradually formed beliefs could reflect their learning processes and effectiveness in the digital learning context [[3], [4], [5], [6]].

Based on Zimmerman's three-phase self-regulated learning (SRL) model [7], people's beliefs on DLPs selection (i.e., forethought phase: task analysis and motivational beliefs) could impact on their learning strategies use (i.e., performance phase: self-control and self-observation), and their justification for their learning outcomes (i.e., self-reflection phase: self-evaluation and self-reaction). Therefore, people's DLPs preference represents the adaptative process between SRL and the features in the DLPs. People's beliefs on their SRL capabilities and their justifications of the features in DLPs are supposed to mutually impact each other and produce lasting impact on their decision on future DLP selections.

Very few studies have taken the perspective of the DLP preferences as a starting point for investigation. Most studies merely applied self-reported questionnaires or instruments to conduct explorations from a quantitative perspective. In the last two decades, to the best of our knowledge, there has been no research to date demonstrating an in-depth picture about the differences in people's DLPs preferences from learners' SRL perspectives of behaviours, cognition, and affection, and how these different types of DLPs preferences were formed based on the learners' previous DL experiences. As the interactions and cooperation between human and technologies becoming sophisticated, we believe that only by better understanding the human factor can we make better use of educational technology.

Therefore, in this study, we focus on investigating learners’ DLPs preferences, with the aim to explore the factors (i.e., self-regulatory behaviours, cognition, and affection) that impact on digital learning choices. For in-depth inquiry, we use a sequential exploratory research approach including a combination of quantitative method (i.e., self-reported choices for clustering), qualitative method (i.e., self-reported interviews for content analysis), and data mining (i.e., sentiment analysis for comparison based on clustering) to provide a comprehensive portrait of learners with different DLP preferences.

RETRACTED

The remaining of this paper is organised as follows. A review of the literature and the knowledge gaps are presented in Section 2. The research method is described in Section 3. Section 4 reports the results of this study. The implications of the findings are discussed in Section 5. Finally, our study limitations and conclusions are presented in Section 6, 7 correspondingly.

## 2 Literature review

### 2.1 Theoretical basis: epistemic beliefs

Epistemic beliefs can act as a lens through which learners interpret and make sense of their DLP preferences [8]. According to Hofer [9], epistemic belief was a multidimensional construct, which consisted of four dimensions of knowledge, i.e., certainty, source, simplicity, and justification. This four-dimension epistemic framework [10] later became the basis for the investigation of Internet-based epistemic beliefs.

Greene et al. [3] and Ferguson et al. [11] developed a three-dimensional framework of Internet-based epistemic beliefs based on the dimension of justification for knowing, comprising personal justification, justification by authority, and justification by multiple sources. Personal justification referred to the extent to which individuals evaluated information found on the Internet based on prior knowledge and reasoning. Justification by authority referred to the extent to which individuals evaluated online information based on the competence and expertise of the resources. Justification by multiple sources referred to the extent to which individuals evaluated online information by checking multiple sources and websites.

In the digital context, with a multitude of digital learning tools to choose from, many factors could impact learners' decisions and reflect their justification for knowing, which varies regarding to their prior digital learning experiences (e.g., tool use, self-regulated learning performance, and the needs for relatedness). In the following sub-sections, we reviewed how previous researchers profiled digital learners’ beliefs and how self-regulated learning features and social features were associated with beliefs.

### 2.2 Profiling digital learners in view of beliefs

Epistemic beliefs were part of learners' profile in online learning [8], but there was a little typology research of DL considering beliefs. For instance, based on Hofer and Pintrich's epistemic theory [10], Lee used self-reported inventory of Internet-based epistemic beliefs to collect data for k-means cluster analysis, revealing four Internet-based epistemic belief groups – the positive beliefs, the negative beliefs, the modest beliefs, and the high justification and uncertainty [12]. However, the authors suggested that interventions or professional training might be necessary for changing students' negative Internet-based epistemic beliefs into positive beliefs, since epistemic ideas might not be relatively fixed and stable beliefs, but were rather more contextually influenced epistemic resources [13]. Therefore, with increasing digital learning experience, people's Internet-based epistemic beliefs could also change.

RETRACTED

In another study, Binali et al. [14] first applied non-hierarchical k-means cluster analysis to classify online learners into five emergent clusters, i.e., highly-engaged self-driven online contributors, moderately engaged self-driven online viewers, less engaged self-driven online learners, highly engaged course-driven online learners, and less engaged course-driven online learners, based on online learning activities, the purpose of online learning, and participants' online learning engagement. Then, these researchers used Scheffe test to compare different groups above based on the three dimensions of justification for knowing, i.e., personal justification, justification by authority, and justification from multiple sources [15]. There found no clear distinct patterns. However, the results indicated that no matter whether the learning was self-driven or course-driven, students who valued justification by multiple sources and justification by authority were more likely to be highly engaged in online learning. It echoes Ferguson and Bråten's opinions [15] that students who had a higher level of knowledge (i.e., those who rely more on justification by multiple sources and authority) might prefer to construct new knowledge through engaging in digital learning.

The two studies above profiled digital learners based on their self-reported Internet-based epistemic belief and online learning behaviours and course features. Very few studies took DLPs beliefs or preferences as a starting point for investigation. Selecting DLPs is a learning process but also a learning product, because the learning product is built up based on people's learning experience and perceptions from the features of DLPs, which would contribute to their DLP beliefs or preferences. The features of DLPs can give people confidence that their learning styles can be satisfied, and their self-regulated learning capacity can be matched.

### 2.3 Self-regulated learning and DLPs beliefs

Self-regulated learning (SRL) is necessary in a self-paced digital learning context. Self-regulatory learners tend to value the learning materials and become more confident in their learning performance in a digital environment [16]. Although previous studies investigated the relationship between epistemological beliefs and SRL [17], self-efficacy beliefs and SRL [18], cultural learning beliefs and SRL [19], almost no studies explore the association between antecedental belief (i.e., DLPs preference) and SRL.

RETRACTED

Muis [6] indicated that epistemic beliefs were activated in the task definition phase of SRL. In other words, digital learners would ponder deeply on how a DLP could contribute to their self-driven learning processes. Different levels of self-regulatory learners performed differently [7]. Such differences may arise even before learners start a digital learning journey, i.e., foreseeing what they are capable of when using certain DLPs that they may have experienced before. Therefore, we assume that justification for learners’ SRL capability is a key component of digital learning beliefs.

### 2.4 DLPs beliefs in social, cognitive, and teaching presence

Self-regulation is not defined as an individualised form of learning because it also includes self-initiated forms of social learning [20]. The need of interactivity in self-driven DL could impact the learners’ choice on DLPs. According to Garrison et al. [21], learning in a distant context occurs at the intersection of social, cognitive, and teaching presence. Social presence refers to the ability of participants to project their individual personalities in order to identify and communicate with the community and develop inter-personal relationships [22]. Cognitive presence refers to the extent to which learners are able to construct and confirm meaning through sustained reflection and discourse [23]. Teaching presence refers to the design, facilitation, and direction of the social and cognitive processes for the purpose of realising the relevant learning outcomes [24].

Recent research calls for the need to investigate the role of learner characteristics in a community of inquiry [8]. Shea and Bidjerano [25] suggested that teaching presence and social presence have a differential effect on cognitive presence, depending upon learner's online self-regulatory learning presence. In the DL setting, learners may keep running into problems and some of them may need an instructor to guide as well as motivate them to solve the problems, or they may wish to have a study group to facilitate the sharing of information and stimulate collaboration (i.e., help seeking). We believe that learners will also evaluate to what extent the features in the DLPs that they are going to select can fulfil their needs in terms of social, cognitive and teaching presence.

RETRACTED

### 2.5 Research gaps

Previous studies have provided insights about classification of digital learners regarding their Internet-based epistemic beliefs [12], the associations between online learning behaviours and the Internet-based epistemic beliefs [14], and the connection between epistemic beliefs and self-regulation in some specific DL context [17], but few studies discussed DLPs preference types in a natural self-driven learning context.

In the face of increasing diverse DLPs, a key question is how different kinds of people holding different kinds of Internet-based epistemic beliefs would adopt different kinds of DLPs. Clarifying the learner typologies regarding DLPs is valuable to educators and instructional designers for their selections of appropriate digital learning platforms, tools, and formats, and to educational policy makers for their strategic decisions on digital learning program investment. Therefore, the first aim of the present study seeks to categorise people with their DLPs preferences. The first research question is:

RQ1 *What distinct learner profiles emerge from people's selection of DLPs?*

Second, almost all the above studies conducted cluster analysis from a quantitative perspective. It is worth clarifying what DL experiences and perceptions construct people's beliefs towards their DLPs selections from a qualitative perspective. Qualitatively investigating people's epistemic justifications toward diversity of digital platforms or tools enables us to comprehend what key features learners are more concerned about. The qualitative results can offer more robust and detailed suggestions for educators and designers. Therefore, the second aim of this study is categorising the key features that people justified from their DL experiences and mapping out the associations among the key features. So, the second research question is.

RQ2 *What dimensions of epistemic justifications emerge from learners' DL experiences and perceptions? And how are these dimensions associated with one another?*

Third, based on the above two aims, our last aim is to qualitatively compare the perceptions of the key features towards digital learning by people of different clusters. This will provide insights on instructional designs that can enhance different learning belief holders’ learning engagement and effectiveness and even change their justifications of knowing from negative perspective to positive perspective. So, the corresponding research questions were formulated as follow.

RETRACTED

RQ3 *What are the differences in the epistemic justification among distinct learner profiles based on their DLP selection?*

## 3 Methods

Almost all previous similar studies were conducted in general context, i.e., using Internet-based epistemic beliefs self-reported instrument to show their associations with other factors such as learning behaviours [14] and self-regulation [17]. However, people could hold different beliefs in different context of DLPs. People's preferences in different DLPs could be reflected on their epistemic beliefs correspondingly. Moreover, merely showing the correlations between DLP beliefs with other factors may not provide a comprehensive understanding on how and why digital learners choose their DLPs. Therefore, a mixed-methods approach that utilised an explanatory sequential design was conducted. This design involves initial collection and analysis of quantitative data and then qualitative data which is obtained to expand the quantitative findings [26], followed by data mining performed for exploring the sentimental differences based on the results of quantitative and qualitative data.

### 3.1 Participants

Convenient sample participants were invited to participate in an online survey during the COVID-19 pandemic in the end of January in 2020. Two authors posted a survey link that was created on an online survey service platform (i.e., wjx.cn) on their personal social media platforms (i.e., WeChat) to call for people to participate.

To snowball our study sample size, the participants were encouraged to share this survey link on their personal social media platform to reach more audiences. After participants completed the online survey, they were also invited to participate in an open-ended survey-based interview. The online survey and interviews were written in Chinese. All the survey participants and interviewees were from China.

As of February 5, 2020, 217 participants completed the online survey. Responses from 16 participants were identified as straightliners and were removed from the dataset. 201 questionnaires were eligible for being analyzed (see Table 1 for survey participants' demographic information). Thereinto, 16 participants voluntarily participated in the open-ended questions (see Table 2 for the interviewees’ backgrounds).

**Table 1:** Demographic background of survey participants.

	Value	Number of participant (percentage)
Total		201 (100%)
Gender	Female	125 (62.19%)
	Male	76 (37.81%)
Age	8–16	2 (1.00%)
	16–24	32 (15.92%)
	24–32	58 (28.86%)
	32–40	39 (19.40%)
	40–48	23 (11.44%)
	48–56	12 (5.97%)
	56–64	33 (16.42%)
	Above 64	2 (1.00%)
Highest degree	Below bachelor	51 (25.37%)
	Bachelor	77 (38.31%)
	Master	55 (27.36%)
	PhD	18 (8.96%)

RETRACTED

**Table 2:** Demographic background of survey interview participants.

No.	Cluster	Gender	Age	Highest degree	Location
#01	3	Female	24–32	PhD	Hong Kong
#02	4	Male	16–24	below Bachelor	Inner Mongolia
#03	1	Male	16–24	Bachelor	Shanghai
#04	1	Female	24–32	Bachelor	Zhejiang
#05	4	Male	24–32	PhD	Guangdong
#06	4	Female	40–48	Bachelor	Shanghai
#07	2	Female	24–32	PhD	Shanghai
#08	1	Male	32–40	Master	Hong Kong
#09	2	Female	24–32	PhD	Guangdong
#10	4	Female	24–32	Master	Beijing
#11	3	Male	16–24	below Bachelor	Shanghai
#12	4	Male	24–32	Bachelor	Hong Kong
#13	3	Male	24–32	Master	Guizhou
#14	1	Female	24–32	Master	Hong Kong
#15	1	Male	40–48	PhD	Shanghai
#16	3	Female	24–32	PhD	Zhejiang

### 3.2 Data collection

#### 3.2.1 Online survey

The online survey consisted of three components: consent form, demographic information (i.e., age, gender, education background, and family monthly income), and DLP choices for a formal learning in a digital context. Before the participants took the survey, we asked for their informed consent to collect their anonymous responses as our data in the opening page. Then they would fill in their background information. Regarding DLP selection, participants were asked to choose (dichotomous choice – Yes/No) the formal approaches for their DL regarding seven common formats available in China.

1. Online learning on MOOC platforms (e.g., Coursera)
2. Online learning through online training institutes
3. Online continuing education through learning management system (LMS)
4. One-on-one private tutoring on social media (e.g., WeChat)
5. Self-organised online learning group on social media (e.g., WeChat)
6. Reading an eBook
7. Mobile learning on educational apps

#### 3.2.2 Open-ended survey for text-based interview

After completing the online structured survey, participants were invited to respond to a list of open-ended questions. The questions were about their digital learning opinions, motivations, experiences and learning perceptions (see the list of questions below). The open-ended questions were only collected once. No follow-up questions were asked based on their responses.

i. What do you think about digital learning or online learning?
ii. Regarding different types of digital learning, do you think some types are more likely to be considered as a formal learning approach than others? Please give an example.
iii. Are there any common feature for those types of digital learning that you think are more formal? Please give an example.
iv. For the knowledge that you want to acquire, does self-directed online learning work for you? Why?
v. Under what kind of situation will you choose digital learning?
vi. In what learning environment do you conduct digital learning? Why?
vii. Do you think you can learn anywhere anytime through digital learning?
viii. Among the different types of digital learning, which one are you most satisfied with? Why?
ix. Among the different types of digital learning, which aspect do you think needed to be improved?

RETRACTED

### 3.3 Data analysis

To answer the three research questions, latent class analysis, qualitative content analysis, and sentiment analysis and comparative analysis were conducted correspondingly.

#### 3.3.1 Latent class analysis

Latent class analyses were performed with participants’ preferences of different types of digital learning pathways. It was considered a person-centred approach that can identify how individuals can be classified according to a set of variables [27]. The person-centred approach was considered more applicable to our purpose, because the aim of the current study was to group people in terms of how they may possibly hold beliefs differently regarding different choices of DLPs (i.e., whether some digital learning pathways work for them as a formal learning approach).

#### 3.3.2 Qualitative content analysis

Based on survey interviewees' responses on the open-ended questions, a qualitative content analysis with conceptual analysis and relational analysis was conducted. Interviewees’ self-reflection on what and how they thought about digital learning experiences and perceptions were analyzed. The unit of analysis was based on completed sentences.

First, the first author reviewed all the survey questions and responses from each interviewee for several times to identify participants’ experiences, opinions, and perceptions towards digital learning. Second, the contents of opinions, experiences, activities, and behaviours that were repeatedly mentioned were coded (i.e., an initial label). Third, after all the contents were coded, the codes with similar meaning would be merged as a concept or an attribute of a concept based on the coding scheme (see Table 3).

**Table 3:** Coding scheme.

Dimension	Sub-dimension	Definition/example
Justification of resources	Justification by authority	Individuals evaluate DLPs based on the competence and expertise of the resources it provided
	Personal justification	Individuals evaluate DLPs based on previous experiences
	Justification by multiple sources	Individuals evaluate DLPs by checking multiple sources and resources
Justification of self-regulated learning (SRL) capability	Self-motivational beliefs	Individuals' beliefs on learning gained through the DLPs
	Learning strategies	Individuals' learning strategies that can be adopted through the DLPs
	Self-evaluation of SRL efficacy	Individuals' confidence on their SRL capability
Justification of social presence	Teaching presence	The design, facilitation, and direction of the social and cognitive processes for the purpose of realising the relevant learning outcomes through the DLPs
	Social presence	The opportunities of the DLPs provided for communicating with the community and develop inter-personal relationships
	Cognitive presence	Ability to construct and confirm meaning through sustained reflection and discourse in the DLPs

Then, a list of codes was created. Forth, conceptual analysis was conducted based on the list of codes to re-code all the contents for a calibration. Fifth, based on the list of codes, we used cognitive mapping to do relational analysis, i.e., two or above concepts that co-occurred in one unit of analysis (i.e., a complete sentence) were mapped to clarify which and how a concept could relate to other concepts. After the qualitative content analysis, a list of key concepts and corresponding attributes was concluded and a cognitive map among these concepts and attributes was figured out. At last, the second author went through all the content and coded segments to evaluate the accuracy of the list of key concepts, affect extraction, and the cognitive map. Two authors discussed the controversial codes to reach a consistent decision.

RETRACTED

#### 3.3.3 Sentiment analysis

For each coded segment above, sentiment analysis was conducted to label them into positive perception, neutral perception, and negative perception. Sentiment analysis enables us to identify the general sentiments expressed in text data. In this study, BytesView data analysis tool (https://www.bytesview.com/) was applied. BytesView is one of the most effective and easiest ways to get quantitative-oriented sentiment result from unstructured text data. It supports multiple languages, including Chinese. For each coded text segment we input, BytesView calculates the percentages of the sentiment perspectives on positive, neutral, and negative through natural language process. Then, the tool will visualise the results on the analytical dashboard to facilitate our interpretation and decision.

Based on the sentiment analysis results from BytesView, the authors went through each text segment again to check the reliability from the perspective of the authors’ perception. For those results we disagreed with BytesView, we would go back to the interview records in order to comprehend the context, and make a final decision through discussion regarding those controversial results between the perspective of machine (i.e., BytesView) and human (i.e., the authors).

The number of interviewees in each key concepts of each sentiment perspective in each cluster was counted. In each cluster, if the number of interviewees held positive perception on one key dimension is larger than the number of interviewees who had negative and neutral perceptions, the interviewees in this key concept would be marked as “positive perception”. On the contrary, if the number of interviewees held negative perception on one key dimension is larger than the number of interviewees who had positive and neutral perceptions, the interviewees in this key concept would be marked as “negative perception”. After all the dimensions of these justifications were marked, the sentiments among these clusters based on the key concepts were compared to clarify the pattern of differences.

RETRACTED

## 4 Results

### 4.1 Distinct learner profiles based on DLPs beliefs

#### 4.1.1 Latent class analysis based on DLPs beliefs

As can be seen from Table 4, the statistics of Bayesian Information Criterion (BIC), Akaike Information Criterion (AIC), entropy, and the Lo-Mendell-Rubin Likelihood Ratio Test (LMR-LRT) were assessed to reflect the model fit. BIC is a measure of goodness of fit that penalises for model complexity [28]. Smaller values of BIC are indicative of better fit. Values of AIC may be interpreted in a similar manner to that of BIC, where smaller values indicate better fit. In making model comparisons, differences in BIC (and AIC) of 10 or more were considered to be very strong evidence of model fit corresponding to the odds of 150:1 [29]. Entropy values indicate the degree to which clusters may be considered distinguishable from one another with standardised values ranging from 0 to 1 [27]. An entropy value closer to 1 indicates the presence of clear, distinct clusters and greater power to predict cluster membership [30]. The LMR-LRT is a test of statistical significance, where the null hypothesis is the number of classes, c, estimated minus one (e.g., H0: c - 1 model fits). For instance, in testing a three-cluster solution (e.g., c = 3), we would reject or fail to reject a two-cluster solution (e.g., c −1 = 3 -1 = 2) using the LMR-LRT statistic. Additionally, the number of free parameters was also reported for each c-class model estimated.

**Table 4:** Statistics of latent class analysis.

	5 groups	4 groups	3 groups	2 groups
Total number of participants (Percentage)	91 (42.72%)	31 (14.55%)	49 (23.00%)	42 (19.72%)
Number of Free Parameters	39	31	23	15
AIC	1441.873	1442.175	1461.824	1492.627
BIC	1572.964	1546.375	1539.133	1543.047
Adjusted BIC	1449.384	1448.146	1466.253	1495.516
Entropy	0.903	0.89	0.785	0.814
Lo-Mendell-Rubin Adjusted LRT Test	0.0373	0.0118	0.2345	0

Above all, four-group clustering was considered the most appropriate result from statistical perspective. The percentage of the participants’ digital learning pathways preferences was shown in Fig. 1. Based on the response distribution on each type of digital learning pathways and corresponding features in each cluster, we defined these clusters as follow:

RETRACTED

**Fig. 1:** Visualization of responses distribution on each item in each group.

**Cluster 1 – Digital learning advocate**: people who prefer to believe that all kinds of digital learning pathways can promote their learning.

**Cluster 2 – Informal digital learner**: people who prefer to learn through asynchronous self-paced learning pathways, such as eBooks reading, mobile educational apps or social media.

**Cluster 3 – Formal digital learner**: people who prefer to have well-designed online courses with systematic learning materials.

**Cluster 4 – Digital learning skeptic**: people who do not have a high preference on any kind of digital learning pathways, in particular for those self-paced informal learning pathways, such as eBooks reading, mobile educational apps, and online group learning on social media.

#### 4.1.2 Chi-Square test on gender, educational background and family income

Chi-Square test for independence had been conducted on the gender, educational background and family income distribution in the four clusters. For gender, it indicated significant association between gender and the clusters, χ2 (3, n = 201) = 10.66, p = .01, Cramer's V = 0.23. The number of female digital learning skeptics was significantly smaller than expected (Adjusted Residual = −3.2), while the number of male digital learning skeptics was significantly larger than expected (Adjusted Residual = 3.2). For educational background, there was a significant association between educational background and the clusters, χ2 (9, n = 201) = 18.53, p = .03, Cramer's V = 0.17. The number of people with secondary education or below in the cluster of digital learning advocate was significantly smaller than expected (Adjusted Residual = −2.4). The number of people with doctor degree in the cluster of digital learning skeptics was significantly larger than expected (Adjusted Residual = 3.0). For family income, there was a significant association between family income and the clusters, χ2 (9, n = 201) = 16.93, p = .05, Cramer's V = 0.17. Thereinto, the number of people with family income between 5k to 10k in the cluster of digital learning advocate was significantly smaller than expected (Adjusted Residual = −2.2), while with the same family income group the number of people in the cluster of informal digital learners was significantly larger than expected (Adjusted Residual = 3.1). For the people in the group of family income between 10k to 30k, the number of people in the cluster of digital learning advocate was significantly larger than expected (Adjusted Residual = 2.6), while the number of informal digital learner was significantly smaller than expected (Adjusted Residual = −2.9).

RETRACTED

### 4.2 Justifications of beliefs on DLPs

Three major justifications of belief on DLPs – justification of resources, self-regulated learning capability, and social presence – were identified based on the qualitative content analysis.

#### 4.2.1 Justification of resources

Online learning resources in our study were judged from three dimensions: personal justification, justification by multiple sources, and justification by authority. ***Personal justification*** referred to learners' information evaluation on ease of use, systematic of resources, and substitute for offline learning etc. ***Justification by multiple sources* referred to learners'** comparative evaluations on the values between recorded resources and live broadcast resources for self-directed learning, and the comparisons of the effectiveness between digital learning and face-to-face learning. *Justification by authority* referred to learners’ evaluation on their learning resources regarding the competence and expertise features that the digital sources enable.

#### 4.2.2 Justification of self-regulated learning capability

Self-regulated learning capability was judged by self-motivational beliefs, digital learning strategies, and general confidence towards self-regulated digital learning. ***Justification of self-motivational beliefs* consisted of learners**’ explicitly knowing their learning motivations and being aware of their learning self-efficacy. ***Justification of digital learning strategies*** meant that learners know what actions they are capable of and can be used to deal with their online learning problems. *Justification of self-regulated digital learning efficacy* meant that learners understand that they are required to have the self-regulatory capability for their digital learning, and they believe they can successfully regulate themselves through the DLPs they choose.

#### 4.2.3 Justification of social presence

Social presence was judged by sense of others, interactions between the instructor and the learner, interactions among learners, and monitoring from the instructor. *Justification of sense of others* referred to learners' perceptions and awareness of other peer learners or instructors in their digital learning environment. ***Justification of interactions among teachers and students*** referred to social behaviours among learners in an online learning environment. ***Justification of the sense of teachers' monitoring* referred to learners**’ awareness of other-regulation for their self-directed digital learning.

RETRACTED

#### 4.2.4 Associations among the justifications

On a macro level, the above justifications were mutually associated (See Fig. 2). More specifically on a micro level, for justification of resources, justification by authority is associated with learners' justification on their self-motivational beliefs and their learning strategy. For instance, the expertise of digital learning resources (e.g., more professional systematic design) can boost target audience’ learning motivations. The feature of the digital learning materials (e.g., recorded materials) is associated with the support for learners' rehearsal strategy. Personal justification about their previous digital learning experiences is associated with the impact on justification of their sense of relationship with online instructors. Justification on multiple sources may reflect learners’ experiences on choosing their DLPs and that should enable a greater sense of social presence for them. For instance, live streaming classes can be a substitute for offline learning because it brings more natural communication and synchronous interactions among the instructor and peer learners.

**Fig. 2:** Cyclical associations among justifications by self-regulated learning capability, sources, and social presence.

Regarding justification of self-regulated learning capability, higher self-motivational beliefs, such as higher self-efficacy on selecting appropriate high-quality digital learning resources, could promote learners' self-instruction strategy. Such higher capability for self-instruction might reflect that learner engaged in more comparisons and evaluations among different digital learning materials (i.e., justification on multiple sources). Perceiving others with the same learning interests could promote intrinsic interactions among online learners. In general, lower confidence in one's SRL capability could indicate that learners might need more monitoring from instructors for their learning processes.

In terms of justification of social presence, online interactions among instructors and learners would impact their justification on their self-regulated learning capability. For instance, instructors' online feedback could improve learners' self-efficacy to participate in digital learning activities. More peer interactions might reveal that more frequency of help seeking learning strategies were conducted. Furthermore, instructors' online monitoring might help to improve learners' general confidence in their SRL capability through others’ regulation in a digital context.

RETRACTED

### 4.3 Different affective perceptions among clusters

As we can see in Table 5, digital learning advocates (Cluster 1) had more positive sentiments than other clusters, while digital learning skeptics (Cluster 4) had more negative sentiments than other clusters. Informal digital learners (Cluster 2) had few positive sentiments, while formal digital learners (Cluster 3) basically had neutral sentiments.

**Table 5:** Comparison of affective perceptions of epistemic justifications among Clusteres

Note. nm: not mentioned. Green highlights: more positive sentiments than neutral plus negative sentiments. Red highlights: more negative sentiments than neutral plus positive sentiments. Gray highlights: no clear preference on sentiment.

Specifically, for justification by social presence, the interviewees in Cluster 1, Cluster 2 and Cluster 4 all held negative perception on the sense of others in the digital learning context. The interviewees in Cluster 3 negatively perceived monitoring from instructors. For Cluster 4, they were also not satisfied the interaction between instructors and learners. For Cluster 2, they held positive perception on peer-to-peer interactions.

For justification by self-regulated learning capability, both Cluster 1 and Cluster 4 interviewees negatively perceived their general SRL capability in digital learning context, but Cluster 1 seemed to have higher efficacy on learning strategies for digital learning.

For justification by resources, it was obvious that Cluster 1 (i.e., digital learning advocates) perceived more positive sentiment on all dimensions. There was no doubt that Cluster 4 (i.e., digital learning skeptics) perceived more negative sentiment on the dimensions of authority and personal justification. Cluster 2 (i.e., informal digital learning) held positive perception on the justifications by multiple sources. Cluster 3 (i.e., formal digital learning) seemed to have no clear preferences on all the dimensions.

## 5 Discussion

### 5.1 Brief summary

This study applied a mixed method to investigate people's different epistemic justifications on digital learning pathways (DLPs). First, a latent class analysis was conducted to categorise digital learners into four groups (i.e., advocate, informal, formal, and skeptical learners) in terms of their preferences on different DLPs. Then, a qualitative content analysis was conducted to categorise digital learners' epistemic beliefs into justifications by digital learning social presence, by self-regulated learning capacity, and by resources. Following that, a relational content analysis was conducted to demonstrate how learners' justification for knowing was associated with or mutually impacted one another. Furthermore, a comparative analysis was conducted based on learners' sentiments on each dimension, elaborating on how different the four groups of digital learning believers justified their digital learning experiences and opinions.

RETRACTED

### 5.2 Profiling digital learners in view of their beliefs on DLP choices

Unlike previous studies that focused on people's justification for knowing and knowledge in a specific digital learning activity [15], this study used peoples' responses of their preferences on a group of DLPs in a general digital learning context. Similar to Lee [12], four groups were revealed in our latent class analysis. Positive believers (i.e., digital learning advocates) and negative believers (i.e., digital learning skeptics) were also found in our study. People with positive digital learning experiences may reflect their positive beliefs on all kinds of DLPs, while people with partially or entirely negative digital learning experiences may resist some or all kinds of digital learning, indicating that people's previous digital learning experiences might influence their choices of DLPs.

Unlike the two other vague clustering results (i.e., modest belief learners and high justification and uncertainty learners) in Lee [12], this study clarified two distinct clusters between the two extremes, i.e., the learners who preferred formal-systematic learning pathways – formal digital learners – and who preferred informal-non-systematic learning pathways – informal digital learners. People's internet-based epistemic beliefs were probably highly associated with their previous digital learning experiences. Based on peoples' personal justification of previous learning experiences, they were more likely to prefer to use those DLPs that they believed could help with their learning. Therefore, the development of enjoyable initial digital learning experiences is important. Non-effective digital learning experiences from a specific pathway might influence learners' perceptions on the extent of knowledge they gained. Less knowledge gaining brought more negative personal justification. Therefore, as an extension of Kintsch's interpretation [31], these learners with fewer gains may not have undergone learning progresses. It does not necessarily mean that they are not capable of constructing new knowledge, but the inappropriate digital learning experiences may prevent them from believing that they have obtained key information to gain new knowledge.

However, according to Ferguson and Bråten [15], we believe that group membership based on belief on DLPs can be malleable, because digital learning decisions depend on learners' justification on their newest digital learning experiences, i.e., learners' digital learning and instructors’ digital learning design are mutually regulated (i.e., co-regulation) from a long-term perspective.

RETRACTED

### 5.3 Social cognitive justifications on digital learning

This study highlighted that the justifications toward digital learning experiences did not merely refer to the justification for knowing which digital learning resources were better or more informative for knowledge construction, but also included people's self-evaluation on their learning capabilities (i.e., knowing about oneself) and the sentiments that the DLPs brought to them (i.e., knowing about the environment). The three dimensions of knowing mutually impact one another, which can be a virtuous circle (i.e., positive impact) or a vicious circle (i.e., negative influence). In summary, people's needs on digital learning are not merely about selecting digital resources. Self-regulated learning capabilities can also highly influence their justifications on other aspects and in turn determine their selection on digital learning pathways.

However, these self-regulated learning capability for most of the time was developed in an offline learning context. For digital learners, they must know what various digital learning pathways can and cannot offer them, and then regulate what they decide to pay effort on. Therefore, the design for nourishing self-regulated learning need to be taken into consideration in the digital learning processes. For instance, the competences of the digital learning resources and the sense of teachers' monitoring were two outstanding demands from the digital learners’ feedback. Digital learning resources are not merely about the content. These digitised contents also need to be enabled more competences, from simply able to be used repeatedly to well-designed personalised learning scaffolding that enable digital learners to be informed about what learning strategies should be used to manage their self-paced learning.

### 5.4 Choices on DLPs reflected on justification for knowing

Unlike [14] investigating peoples' justifications on digital learning from the behavioural perspective, this study used mixed method from both quantitative and qualitative perspectives and found that peoples’ belief preferences on different digital learning pathways did reflect their different justification in terms of digital learning resources, their SRL capability, and social presence in the digital learning context.

Although Cluster 1 (i.e., digital learning advocates) seemed to accept all kinds of digital learning platforms, these learners might still not have positive social presence, especially for the sense of others like in a face-to-face learning setting.

RETRACTED

Similar to Cluster 1, Cluster 2 (i.e., informal digital learners) were those who probably had higher self-regulated learning capability but were also unsatisfied with the intensity of the sense of others in digital learning. However, Cluster 2 learners positively perceived their interactions with peers. It may be because informal learners used social-media-style applications, such as mobile educational apps or other commercial digital products. Heavily depending on social networks may have strengthened their online interaction with other people, no matter the interactions are synchronous or asynchronous.

Cluster 3 (i.e., formal digital learners) were those who were likely to have low self-efficacy on their self-directed learning. That is why these learners might have higher level of requirements regarding teachers’ monitoring, because they needed formal and professional support from instructors in a formal learning setting, such as a well-designed systematic online course on Coursera.

Cluster 4 (i.e., digital learning skeptics) were those who negatively or less positively perceived epidemic beliefs on digital learning. These learners were not confident in their self-regulated learning in general, and they did not trust the digital learning resources to be as well-designed as offline face-to-face class in terms of the professional level of instructions. Similarly, they were also less likely to believe that these DLPs could bring social presence for them like in a face-to-face class. For these learners, online instructors may need to take external motivational design components into the DLP in order to improve their digital learning experiences, and then may change their beliefs in future.

Overall, the preferences of the choices on DLPs were based on learners' epistemic beliefs toward their digital learning, which was constructed by their previous digital learning experiences. However, even though they were labelled as one cluster, these learners’ decisions on digital learning were malleable by calibrating their justifications on themselves, the resources, and the environment for digital learning. Such variety in requirements suggests that digital learning instructional design should be further explored to consider how to better fit the learning expectations of different kinds of people in different types of learning pathways learning various kinds of contents.

## 6 Limitations

This study has some limitations that should be considered. First, data analysis could be slightly biased due to our convenient sample with only Chinese cultural backgrounds, even though the sample size was large enough to support the quantitative analysis. Future study can consider recruiting participants from other cultural background for the clustering analysis and compare the results to this one. Second, the data was collected during the COVID-19-relevant school suspension and city lockdown. Therefore, people's responses to our items and interviewees may be influenced by the situations of working at home or home schooling. As the epidemic subsides, a follow-up study can be conducted without the effects of the epidemic to investigate the changes. Third, although the interviewees were matched samples with our survey participants, the number of participants in each result cluster was too small for drawing a robust comprehensive conclusion. Future studies are suggested to conduct a more in-depth interview study built on the qualitative findings of this study. In addition, the study can use a validated Internet-based epistemic belief instrument or develop a new digital-learning-based epistemic belief instrument to conduct the quantitative analysis in future.

RETRACTED

## 7 Conclusions

### 7.1 Summary of results

Few studies have taken learners' digital learning pathways (DLPs) preference as a starting point of in-depth exploration from the perspectives of behaviours, cognition, and affection. This study therefore applied a mixed-methods exploratory sequential design to investigate the categories of digital learners regarding their beliefs on DLPs. First, from a quantitative perspective of DLP choices preferences, four clusters, i.e., digital learning advocates, informal digital learners, formal digital learners, and digital learning skeptics, were identified using latent class analysis. Second, from a qualitative perspective of follow-up interviews, three dimensions of justification for knowing were categorised based on content analysis from a small group of survey participants, i.e., justification by self-regulated learning capability on self-motivational beliefs, learning strategies, and general confidence regarding SRL; justification by resources from the perspectives of authority, multiple sources evaluation, and personal experiences; justification by social presence on teacher monitoring, interactions among instructors and peers, and sense of others. A cognitive map based on the three major dimensions of justification for knowing was constructed through relational content analysis, indicating their mutual associations among each other. Third, from the affective perspective of sentiment analysis, no matter quantitative or qualitative analysis, the results revealed that learners in four clusters demonstrated their epistemic justifications differently. Finally, we can conclude that people's digital learning shows differences in behaviours (i.e., DLP choices), cognition (i.e., epistemic justification about digital learning), and affection (i.e., satisfactory feeling about their choice and self-directed learning process).

RETRACTED

### 7.2 Implications

Theoretically, DLP preference is a stage of the digital learning process, and it is also a product of digital learning experiences. Digital learning experiences are not merely constructed from the perceptions about the design of DLPs, but also from learners' justification for knowing about their learning capabilities and social needs. Positive previous digital learning experiences build up learners’ positive justification for knowing about future digital learning choices, whereas negative experiences may exert negative influence on it. Changes in digital technologies could create new needs in learners. In turn, the new needs could pose new requirements for digital learners.

Practically, for digital learning designers, our study suggests them to consider digital learners' epistemic justification on their self-regulated learning processes, social presence and resources, as these could inform designers about learners' individualised needs. For instructors, our study informs them to take both formal and informal features of DLPs into account to meet various digital learners' preferences. For policy makers, teachers’ professional training on digital teaching should be promoted to improve their digital literacy, which is essential for creating new and suitable pedagogy in the digital context. For learners per se, this study stresses that the core of the effective digital learning is the self-regulatory learning capability. Learners need to clearly identify their learning needs and goals. Some digital learning strategies, such as environmental structuring and task strategies, should be equipped. Furthermore, integrating design of self-regulatory processes into DLPs should be collaboratively promoted by designers and education researchers.

### 7.3 Future studies

Our study has explored the types of people's DLP preference, the themes of people's epistemic justifications on digital learning, and their affective differentiations in terms of epistemic justifications in different DLP preferences. However, several aspects can be further investigated. First, more in-depth qualitative studies can explore other dimensions of learners' epistemic justifications. For instance, case studies can be conducted in a specific DLP to comprehend how people's DLP choice and their learning processes impact each other. Second, DLP preferences and the learners' epistemic justifications in different instructional context, e.g., blended learning, can be explored and discussed. Third, with artificial intelligence (AI) developing, researchers can try to identify learner's epistemic justifications with the help of AI and to provide instant individualised DLPs.

RETRACTED

## Author contribution statement

Min Lan: Conceived and designed the experiments; Performed the experiments; Analyzed and interpreted the data; Contributed reagents, materials, analysis tools or data; Wrote the paper.

Qian Huang: Analyzed and interpreted the data; Contributed reagents, materials, analysis tools or data; Wrote the paper.

## Funding statement

This work was supported by the National Social Science Foundation of China, Youth Project in Education. The project is titled "Action Research on Optimising Teachers' Online Instructional Design from the Perspective of Regulation Theory" [Project No. CCA220320].

## Data availability statement

Data will be made available on request.

## Additional information

No additional information is available for this paper.

## Ethics statement

Ethics approval for the study was obtained from the University of Hong Kong. The approval number was EA1604035.

## Declaration of competing interest

The authors declare that they have no known competing financial interests or personal relationships that could have appeared to influence the work reported in this paper.
